The article "A Systematic Review and Meta-Analysis of the Associations between Immigration Status and Stroke Incidence and Mortality" was published in 2022. Journal: Biomed Res Int.

# A Systematic Review and Meta-Analysis of the Associations between Immigration Status and Stroke Incidence and Mortality

**DOI:** 10.1155/2022/1926744

**Published:** 2022-08-26

**Authors:** Jun-zhen Chen, Hai-mei Wang, Wenhao Zhu

**Affiliations:** ^1^Department of Encephalopathy, Zibo Hospital of Traditional Chinese Medicine, Zibo, Shandong 255300, China; ^2^Department of Oncology, Zibo Central Hospital, Zibo, Shandong 255300, China

## Abstract

**Methods:**

We thoroughly searched PubMed, Embase, and MEDLINE databases for the literature on stroke risk for immigrants and host populations by January 2022. Fourteen relevant cohort studies from eight countries met the inclusion criteria, and their data were included in this meta-analysis. Heterogeneity and publication bias were assessed.

**Results:**

The results showed that the immigrant groups suffered from a lower incidence rate of stroke compared with the host populations (HR = 0.81, 95% CI 0.71–0.91, *P* = 0.001), but there was nonsignificant higher mortality of stroke in immigrants (HR = 1.07; 95% CI 0.84–1.36). However, the pooled adjusted incidence HR reduced to 0.67 (95% CI 0.60–0.75) after adjustment for publication bias. Immigrants had a lower stroke incidence compared to long-term residents, but the association varied with the country of origin, socioeconomic status, residence (urban *vs.* rural), and comorbid conditions. *Discussion*. The present systematic review and meta-analysis implicated that stroke risks are different for immigrants and the host populations; therefore, this knowledge may be useful for developing targeted stroke prevention strategies.

## 1. Introduction

Large-scale immigration has remained one of the great human activities for the past 100 years. According to the United Nations report on international migration, 3.4% of the world population represent international migrants, while 14% of the population in high-income countries are immigrants [1]. Europe (82 million people) and North America (59 million people) are the areas with the largest immigrant population in the world, and these numbers are expected to rise in the next few decades [2, 3]. The Global Burden of Disease, Injuries, and Risk Factors Study (GBD 2010) has estimated that stroke was the second most common cause of death and the third most common cause of disability-adjusted life-years (DALYs) in the world [4, 5]. Globally, stroke is the main cause of death, prolonged hospitalization, and long-term disability of patients, seriously affecting the quality of life and causing a heavy burden to society and families, while recurrent patients are even at a greater risk of death. Studying the stroke differences between immigrants and the host population can be a potential source of insight into the causes of illnesses and their prevention and treatment. These differences are largely attributed to a wide variety of pre- and postimmigration demographic, socioeconomic, ethnic, cultural, biological, and behavioral factors of these immigrants [6]. Identification of the stroke risk difference between immigrants and the native regarding the relevance between immigration status and stroke occurrence and prediction of the risk of disease occurrence has not only been a global but also a clinical concern in need of timely scientific research [6, 7].

This review is aimed at identifying the patterns of stroke risks among immigrants from high-income countries in Western Europe and North America and how the risk of stroke varies with the country of origin. The second objective was to assess the influencing factors related to stroke among immigrant groups in the host countries.

## 2. Materials and Methods

### 2.1. Literature Search

This study used the method of Hai-mei Wang et al. [8], and the description of the methods partly reproduces their wording. The present study was rigorously designed and reviewed according to the guidelines of the Preferred Reporting Items for Systematic Reviews and Meta-Analysis (PRISMA) statement checklist [9–11]. This systematic review and meta-analysis was registered (PROSPERO registration no. CRD42022306377) online. PubMed, Embase, and MEDLINE were comprehensively searched for eligible studies up to January 2022. With the language limited to English, we included the following keywords to search for the relevant literature: “immigrant OR “emigrants and immigrants” OR “emigration and immigration” OR migrants OR migration” AND “stroke OR cerebrovascular accident OR cerebral infarction OR cerebral embolism OR ischemic stroke OR subarachnoid hemorrhage OR intracerebral hemorrhage.” Literature published from 2000 to 2022 was included to capture the most recent information. Additionally, the citation lists of these retrieved articles were manually screened to ensure the sensitivity of the search strategy [8].

### 2.2. Inclusion and Exclusion Criteria

Inclusion criteria were as follows. (a) Studies included in this review were limited to peer-reviewed cohort or case-control studies with sample sizes of at least 1000. The studies we included reported the incidence, mortality rate, or relative risk of stroke in specific immigrant groups or in immigrants overall compared with the host population. (b) Only studies with verified immigrant identities based on the country of birth, immigration records, or in combination with other measures were included. The study population only included first-generation immigrants, regardless of their offspring. (c) Host populations were limited to North America, Europe, and Australia because these regions include the most high-income countries and have a large population of immigrants. (d) We included studies adopting the WHO definition of stroke, which set up standard methods for diagnosing stroke cases and distinguishing stroke subtypes, and those studies in which the final diagnoses of stroke were based on the results of at least one of the following tests: brain imaging, cerebrospinal fluid analysis, or autopsy.

Exclusion criteria were as follows. (a) The results of refugee studies were not presented in this study due to its small population, as factors affecting this group are too complex and distinct from those of immigrants for economic or family reasons. (b) We excluded people not registered with the provincial health insurance plan (visitors, seasonal migrant workers) to exclude transient residents for whom follow-ups are available. (c) Duplicate publications or repetitive analyses were excluded. (d) Reviews, letters to the editor, and abstracts were also excluded.

### 2.3. Data Abstraction and Quality Assessment

All relevant articles were evaluated and extracted by two independent authors (JZC and HMW). Any disagreements were consulted with the third investigator (WHZ). For each study, the following items were extracted from the articles: first author, year of publication, the country of origin, the country of destination, the population size, age range, the range of study years, outcome measures, and the relevant influencing factors, such as marital status, income, residence (urban *vs.* rural), current smoking, and comorbid conditions between immigrant status and stroke. At the same time, WHZ confirmed the accuracy of the extracted relevant information. When more than one HR was reported, the most adjusted HR would be extracted [8]. The extracted HRs and 95% confidence intervals (CIs) were standardized into the form of immigrant groups *vs.* the host populations. Due to the low overall risk of stroke among migrant populations in the included literature, HRs in the cohort studies were mathematically similar to the relative risks (RRs) and odds ratios (ORs) in the cohort studies [8]. Therefore, if the results of RR ratios were provided in the studies, multivariate analysis results would be extracted prior to that of univariate analysis. If a certain study only provided the RR ratios for immigrants from different countries of origin separately, we would calculate the pooled HRs and 95% CIs through indirect extraction. If data of interest were not accessible, we would obtain the missing data from the corresponding authors of included articles [8]. Since all studies included in our meta-analysis were cohort studies, the Newcastle-Ottawa Scale (NOS) was used to assess the quality of each by two independent authors (JZC and HMW). The NOS consists of three parts: selections, comparability, and measurement of outcomes [12]. Studies with NOS scores of ≥6 were marked as high methodological studies. We used part of the methods in our previously published article and quoted it correspondingly in the text.

### 2.4. Statistical Analysis

Stata SE12.0 and RevMan 5.3 software were used for statistical analysis. Pooled HRs and 95% CIs were obtained from the included studies. HRs for incidence, mortality, and ORs for participant covariate parameters were statistically analyzed. Chi-square-based *Q* test and *I*^2^ statistic were performed to assess the heterogeneity of the included trials. If *I*^2^ was >50% or the *P* value was <0.05, significant heterogeneity would be observed, and the random-effects model would be applied. Otherwise, the fixed-effects model would be adopted. Publication bias was evaluated by Egger's test and visual inspection of Begg's funnel plot [8]. The stability of the results was testified by sensitivity analysis [13].

## 3. Results

### 3.1. Study Selection and Study Characteristics

A total of 3320 relevant articles in conformity with our search strategy were retrieved through the database search. After the removal of duplicates, 2840 remaining publications were screened for their titles and abstracts, and 2799 publications were further excluded as they were reviews, letters to the editor, and meeting abstracts or had irrelevant contents. The full texts of the remaining 41 publications were further examined, and 27 publications inconsistent with the inclusion criteria were removed. Ultimately, 14 studies [1, 14–26] were included in this systematic review and meta-analysis. The selection process is summarized in the flow diagram (Figure 1).

The included articles were published between 2000 and 2022. As shown in Table 1, all included articles were cohort studies, with two studies from Denmark [15] and Northern Ireland [20] adopting a prospective method and the remaining 12 using retrospective methods. Four of the studies (28.6%) were conducted in Canada, two (14.3%) were conducted in Sweden, two (14.3%) were conducted in the United States, two (14.3%) were conducted in the Netherlands, and one (7.1%) was conducted each in Denmark, Ireland, Australia, and Portugal. All demographic data investigated were retrieved from the provincial administrative databases, such as the National Patient Registry and the Ministry of Immigration. All studies except one from Sweden [17] were adjusted for confounders, although the variables chosen for adjustment varied. We also compared the hazard of mortality and incidence between immigrants and long-term residents. All studies stratified immigrants according to country or region of birth, except one from Canada [1], one from the United States [26], and one from Sweden [17], which lacked information on ethnic background or country of birth of subjects. Two studies from Sweden [25] and Canada [1] were also stratified on the basis of stroke subtypes of the included population. Among 14 included cohort studies, seven (50.0%) were conducted to study mortality, eight (57.1%) focused on incidence, and one (7.1%) compared the risk of vascular disease recurrence. Two studies (14.3%) from Canada and Denmark simultaneously assessed the outcome of incidence and mortality. The authors, host country, year of publication, study period, and age range of the included population for the two studies were almost identical; thus, the possibility of overlapping patients could not be ruled out. However, we still included the two articles in our research because one focused on the study of the mortality and recurrence rate of stroke, while the other focused on the incidence of stroke.

### 3.2. Incidence Rate of Stroke among Immigrants Compared with That of the Host Populations

Eight studies investigated the incidence rate of stroke among immigrants compared with the host populations. There was significant heterogeneity in these studies (*I*^2^ = 92.4%, *P* < 0.001); therefore, the random-effects model was used to calculate HR and 95% CI. The results showed that migrant groups had a lower incidence rate of stroke compared with the host populations (HR = 0.81, 95% CI 0.71–0.91), which was statistically significant (*P* < 0.01). An estimated 92.4% of the total variability (*I*^2^) in the pooled HR was due to the heterogeneity between studies rather than by chance (Figure 2(a) and Table 2).

### 3.3. Association between Immigration Status and Mortality in Patients with Stroke

Seven studies provided suitable data for mortality analysis. The random-effects model was applied to analyze pooled HR and its 95% CI since apparent heterogeneity was observed (*I*^2^ = 94.5%, *P* < 0.001). As shown in Figure 2(b) and Table 3, the results indicated that the mortality hazard was higher but not significantly different in migrant groups (HR = 1.07; 95% CI 0.84–1.36) compared with that of the host populations.

### 3.4. Subgroup Analysis of the Association between Immigration Status and the Incidence Rate of Stroke according to Country of Origin

According to the world region of origin, we conducted stratified analyses to confirm the relationship between immigration status and incidence rate in patients with stroke in different subgroups. As shown in Table 4 and Figure 3, two of the subgroup analyses, including Eastern and Middle European (HR = 1.02, 95% CI 0.86–1.20, *P* = 0.831) and Latin American (HR = 1.08, 95% CI 0.95–1.23, *P* = 0.257), generated results different from the predictive value of HR between immigration status and the incidence of stroke, yet this difference was not statistically significant. Immigrants from Eastern Europe, Middle Europe, and Latin America might have a higher risk of stroke than the host population. There was no statistically significant difference in the incidence rate of immigrants from developing and transitioning economies and host populations (HR = 0.91, 95% CI 0.79–1.06, *P* = 0.230). Immigrants from developed countries were significantly less likely to be diagnosed with stroke than native people (HR = 0.83, 95% CI 0.74–0.94, *P* = 0.003). Therefore, we considered that the different regions of immigrants' origin might be one of the main reasons for the high heterogeneity of our pooled results.

### 3.5. Association between Migrant Groups and Covariate Parameters

The association between migrant groups and covariate parameter ORs and their 95% CIs were utilized to investigate the correlation between immigration status and baseline characteristics of stroke, including gender, age, follow-up duration, marital status, income, residence (urban *vs.* rural), smoking history, hypertension, diabetes, and dyslipidemia. The results of these analyses are presented in Table 5 and Figure 4. From the pooled ORs, notably significant associations were detected between migrant groups and follow-up duration (OR = 0.68, 95% CI 0.67–0.69, *P* < 0.001), income (OR = 2.13, 95% CI 1.65–2.76, *P* < 0.001), residence (OR = 4.59, 95% CI 3.54–5.95, *P* < 0.001), and hypertension (OR = 1.30, 95% CI 1.08–1.57, *P* = 0.006). Overall, immigrants had a relatively low income. Immigrants suffered from a lower prevalence of hypertension and all migrant populations tended to be more concentrated in urban centers.

### 3.6. Sensitivity Analysis

Sensitivity analysis was conducted by removing each eligible study to test the stability of the pooled result of the association between immigration status and incidence rate in patients with stroke. As demonstrated in Figure 5(a), when “Farhad 2004” [25] was removed, the pooled result fluctuated. Subsequently, recalculation of the pooled HR after removal of “Farhad 2004” showed a similarly lower rate of stroke in immigrants compared to long-term residents (HR = 0.77, 95% CI 0.69–0.85, *P* < 0.001). This means that the significance of the pooled result was not altered by the removal of an eligible study. Therefore, our pooled result was proven to be reliable.

### 3.7. Publication Bias

For the meta-analysis of the association between immigration status and incidence rate in patients with stroke, Begg's funnel plot and Egger's regression test were performed to test for publication bias. Publication bias was evident based on asymmetry in Begg's funnel plot (Figure 5(b)) and the result of Egger's regression test (*P* = 0.024). After that, “Trim and Fill analysis” was adopted to evaluate the influence of publication bias, as previously described [27]. As depicted in Figure 5(c), the adjusted HR (95% CI) was 0.67 (0.60–0.75) (*P* < 0.001), indicating that the publication bias did not have a significant influence on the pooled result; thus, our result was credible.

## 4. Discussion

To the best of our knowledge, a meta-analysis of relative risk for stroke has not been performed in immigrants, and this is the first meta-analysis of the risk of stroke in immigrants. A previous systematic review about the risk of ischemic heart disease and stroke by Sohail et al. [28] is different from our current study in the following aspects. First, the target diseases in Sohail et al.'s research were ischemic heart disease and stroke, while our research involved only stroke, narrowing down the research scope and increasing the accuracy. Second, five studies conforming to inclusion criteria were included in Sohail et al.'s research, including four cases of stroke incidence and one case of mortality. The literature included was published from 2004 to 2014. In our current study, 14 papers were included, and the date of publication was extended to 2021, covering eight studies of stroke incidence and seven studies of mortality. In contrast, we collected a larger sample size and more updated literature, ensuring more comprehensive and updated information, with which more reliable findings could be made. Third, Sohail et al. have only conducted a qualitative systematic review, and there have not been enough studies for a quantitative meta-analysis. Our study conducted a qualitative and quantitative analysis of the incidence and mortality risk of stroke in the migration populations; thus, the findings were more meaningful. In this large population-based cohort study, new immigrants had about a 20% lower relative risk of stroke than the host population, and this was the case for all stroke subtypes. Interestingly, although immigrants from most parts of the world had a lower risk of stroke, most immigrants seemed to have a worse prognosis. Our systematic review and summary of the available published studies regarding the changes in the epidemiology of stroke among immigrants in North America, Western Europe, and Australia established that the incidence of stroke among migrants was much lower than that in the host population (HR = 0.81, 95% CI 0.71–0.91, *P* = 0.001), but there was nonsignificantly higher mortality of stroke in migrants (HR = 1.07; 95% CI 0.84–1.36). Immigrants had a lower incidence of stroke compared to long-term residents, but the association varied with the country of origin, socioeconomic status, residence (urban *vs.* rural), and comorbid conditions. In the individual studies reporting on risk factors for stroke, we found that immigrant groups were less likely to develop stroke if they came from developed countries. We also found that most of the immigrant groups had relatively insufficient income, lower incidence of hypertension, and gathered more in urban areas [29].

In 2019, 272 million people worldwide were international migrants. Europe (82 million) and North America (59 million) are world leaders in accepting immigrant populations, and these numbers are expected to rise in the coming decades [2, 3]. Our meta-analysis results showed that immigrants tend to have better health than the host population because of the “healthy migration effect” [30, 31]. That means that those who are healthy are more likely to migrate. Furthermore, as influenced by American immigration policy, the medical examination required all potential immigrants to be examined to exclude unhealthy candidates [28]. Another hypothesis is the so-called “salmon bias effect,” an expression first used by Pablos-Mendez to describe “the compulsion to die in one's birthplace” [32]. This assumption asserts that many immigrants return to their country of origin when they expect to die shortly [33–35]. If the deaths occurring in their country of origin are not registered in the mortality statistics of the country of residence, the mortality rate of immigrants will be artificially reduced [32–34, 36]. Thus, the “salmon bias effect” indicates that migrants in poor health return to their countries of origin, thereby improving the health profile of migrant cohorts. The country of migrants' origin has also been closely related to ethnic, cultural, and biological factors [37]. Preexisting conditions of patients are closely related to stroke occurrence and prognosis. The higher the risk level is, the greater the degree of intervention is required. Different risk factors have different impacts on stroke [38]. Hypertension is not only a risk factor for the primary prevention of ischemic stroke but also one of the most important vascular risk factors for secondary prevention [16]. Our research showed that the immigrants' risk factors for incidence of stroke, such as hypertension and metabolic syndrome, were relatively less frequent; hence, the risk of stroke for them was lower. We found a smaller proportion of men, a smaller number of married or cohabiting population, fewer history of hyperlipidemia and smoking, and a higher risk of diabetes in immigrants, although these differences were not statistically significant. Even though the overall incidence rate of stroke in migrants was lower than that in the host population, the risk of stroke in migrant groups from Eastern and Middle Europe (HR = 1.02; 0.86–1.20) and Latin America (HR = 1.08; 0.95–1.23) was relatively higher, which is in line with the higher risk of hyperlipidemia events observed in these countries [39–41]. This suggests that when immigrants originate from these countries, we might not be able to observe the “healthy migration effect.” Noteworthily, the experience of immigrant groups from the Caribbean, Baltic State, former Yugoslavia, former Soviet Union, Hungary, and Latin America might be different from that of immigrant groups from other regions. However, our study could not verify if factors, such as discrimination or systematic racism, were the important drivers of these differences in healthcare and outcomes [41–43]. In the future, we can use relevant cultural adaptation measures to assess the health outcomes of immigrants, such as language or education before arrival, time proportion in the destination country, and other factors, such as the number of nonimmigrant friends or other self-reported cultural adaptation scales [44–47]. Unlike patients with chronic diseases, such as cancer, or patients with diseases treated in outpatient clinics, such as cough, patients with stroke usually require symptom evaluation and prompt hospitalization [21]. Therefore, choices of different medical services between immigrants and host populations might also lead to different outcomes of stroke mortality [48, 49].

Key strengths of our study include the originality and initiative of this research topic, as it is the first review in this aspect. Certainly, this study also has some limitations. Our findings might be affected by changes in study sample sizes and follow-up time, both of which can affect the statistical significance of the pooled results [50]. In our review, we found that Europe conducted more comprehensive immigration research than North America and Australia. More comprehensive immigrant cohort studies in North America and Australia are also needed. There is a lack of stratified analysis of residence duration, stroke subtypes, and intergenerational differences, which biases the discussion of the factors that might influence the research results. The larger the sample size and the longer the follow-up time is, the higher the evidence intensity of outcomes observed in high-quality studies will be. Due to the characteristics of stroke, the biggest challenge of follow-up research over time is the loss of follow-ups. Only a small number of the studies we included simultaneously reported mortality, recurrence rate, and disability rate. Therefore, our study also lacks a specific analysis of disability and recurrence rate of stroke. Furthermore, the incidence rate of stroke in some immigrant groups was lower, but the survival time after events was also lower. It is difficult to associate prompt hospitalization and professional care with mortality [51, 52]. Finally, although there are a few representatives of the host country, the studies included in this meta-analysis represented various social and political cultures with different medical systems; thus, the study had relatively large heterogeneity. Future studies on the relationship between migration and stroke risk should include more detailed information on the region of immigrants' origin and the cultural background of the control group. Comparing the host population with immigrants of the same ethnic background will help to control potential genetic differences between ancestral groups and help identify differences in specific cultures and regions [53]. Since Asia is also one of the regions with the largest number of international immigrants in the world, the situations in Asia should also be investigated, as has been done with the European and North American countries, to verify if the results agree with our current research findings.

In conclusion, the results of this study confirmed that there are differences in stroke risk between immigrants and the host population, and the incidence of stroke in immigrants is lower than that in the host population. The size of this gap varies with the place of immigrants' birth, depending on the region, economic status, comorbidity status, living environment, etc. Meanwhile, there might be the impact of barriers, such as medical care, in immigrant populations, which ultimately affects the survival rate. This knowledge might be useful for developing targeted stroke prevention strategies [54].

## Figures and Tables

**Figure 1:** Flow diagram of the study selection process.

**Figure 2:** (a) Forest plots of studies evaluating the incidence of stroke among immigrants compared with the host populations. (b) Forest plots of studies evaluating mortality of stroke among immigrants compared with the host populations.

**Figure 3:** Forest plots evaluating the stratified analyses for the pooled HRs according to country/region of origin regarding a subgroup, including (a) Western Europe, Australia, and North America, (b) Eastern and Middle Europe, (c) East and Southeast Asia, (d) Western Asia/Arab countries, (e) Latin America, and (f) Africa.

**Figure 4:** Forest plots evaluating the relationship between immigration status and participant characteristics, including (a) gender, (b) age, (c) follow-up duration, (d) marital status, (e) income, (f) residence, (g) current smoking, (h) hypertension, (i) diabetes, and (j) dyslipidemia.

**Figure 5:** (a) Sensitivity analysis of pooled HR in patients with stroke. (b) Begg's funnel plot for the association between immigration status and stroke incidence. (c) Funnel plot of “Trim and Fill analysis” (the trim and fill adjusted HR = 0.67, 95% CI 0.60–0.75, random-effects model).

**Table 1:** Baseline characteristics of studies on stroke among immigrants and the host populations.

Host country	Year	Age (years)	Study population size	Source of data registrations for stroke/immigrants	Study period	Study design
Canada [14]	2021	18–104	Long-term residents 31918; immigrants 2740	Ontario Stroke Registry (OSR) and provincial administrative databases (the Ministry of Immigration, Refugees and Citizenship)	2002–2018	Retrospective cohort study
Denmark [15]	2016	≥18	Danish-born 8746; 70339 family-reunified immigrants	The National Patient Registry and the Danish Immigration Services	1993–2010	Prospective cohort study
Canada [16]	2015	30–74	5.2 million long-term residents; 824662 immigrants (from 201 countries of birth)	Citizenship and Immigration Canada's Permanent Resident database and 9 population-based health databases	1985–2000	Retrospective cohort study
Sweden [17]	2014	≥16	321407 Swedish and 307174 foreign-born persons	Statistics Sweden (SCB) and the National Board of Health and Welfare Centre for Epidemiology	1970–1999	Retrospective cohort study
The Netherlands [18]	2014	≥30	Ethnic Dutch 2271489; immigrants 125957 (5 countries)	Dutch national registers: Population Register, Hospital Discharge Register, Cause of Death Register, and Regional Income Survey	1998–2010	Retrospective cohort study
United States [19]	2012	≥50	Non-Hispanic White 14360; foreign-born Hispanic 746	The Health and Retirement Study (HRS)	1998–2008	Retrospective cohort study
Northern Ireland [20]	2011	25–74	Northern Ireland 837646; immigrants 92573	NISRA	2001–2007	Prospective cohort study
Canada [21]	2021	18–104	All immigrants 1216557; long-term residents 6873967	ICES (the Institute for Clinical Evaluative Sciences) and the Immigration Refugee and Citizenship Canada database	2003–2018	Retrospective cohort study
Australia [22]	2011	NA	Australian-born 331483 and immigrants 1275463	Australian Bureau of Statistics (ABS) census data	2001–2002	Retrospective cohort study
Canada [1]	2010	16–65	Long-term residents 3272393; immigrants 965829	Three provincial healthcare administrative databases and the Canadian Institute for Health Information Discharge Abstract Database (DAD)	1995–2007	Retrospective cohort study
The Netherlands [23]	2009	NA	Ethnic Dutch 38489; immigrants 4723	The national hospital discharge register (HDR), the Dutch population register (PR) and the causes of death register of statistics Netherlands	1997–2000	Retrospective cohort study
Portugal [24]	2008	25–64	Born in Portugal 5093910; African migrants 261970	The Instituto Nacional de Estatı'stica in Portugal and tabulated population data from the 2001 Census	1998–2002	Retrospective cohort study
Sweden [25]	2004	40–89	Swedish-born 98961; immigrants 14701	The National Swedish Census investigation and the STROMA	1990–2000	Retrospective cohort study
United States [26]	2010	≥35	Long-term residents NA; immigrants 4943041	The New York City Department of Health (NYCDOH) and US Census Public	1990–2002	Retrospective cohort study

**Table 2:** Summary of results from studies comparing the incidence rate of stroke in immigrants (according to country/region of origin) *vs.* the host population.

Host country	Western Europe, Australia, and North America	Eastern and Middle Europe	East and Southeast Asia	Western Asia/Arab countries	Latin America	Africa
Denmark	Western incl. EU (0.56; 0.42–0.74)	Former Yugoslavia (0.76; 0.68–0.82)	Thailand: NA	Afghanistan (0.71; 0.54–0.93); Iraq (0.73; 0.62–0.86); Turkey (0.77; 0.58–1.02)		Somalia (0.49; 0.38-0.64)
Canada	White-Western European (male) (0.9; 0.8–1.1); white-Western European (female) (0.7; 0.6–0.8)	White-Eastern European (male) (1.3; 1.1–1.5); White-Eastern European (female) (0.8; 0.7–0.9)	(Male) East Asian (0.7; 0.6–0.8); Southeast Asian (1.5; 1.3–1.7); South Asian (1.2; 1.1–1.3) (Female) East Asian (0.6; 0.5–0.7); Southeast Asian (1.0; 0.8–1.1); South Asian (0.8; 0.7–0.9)	West Asian/Arab (male) (0.8; 0.7–0.9); West Asian/Arab (female) (0.7; 0.6–0.9)	Latin American (male) (1.3; 1.1–1.6); Latin American (female) (1.1; 0.9–1.2)	Black (male) (1.5; 1.3–1.8); black (female) (1.1; 1.0–1.3)
The Netherlands			Indonesia (1.03; 0.95-1.12)	Turkey (0.95; 0.81-1.11); Morocco (0.37; 0.24-0.57)	Suriname (1.36; 1.20–1.55); Netherlands Antilles (1.35; 1.01–1.81)	
United States	Hispanics (0.76: 0.55–1.05)					
Australia	North America (0.92; 0.57-1.40); Northern Europe (0.91; 0.33-1.97); the United Kingdom and Ireland (0.65; 0.56-0.75); Western Europe (0.85; 0.68-1.07)	Eastern Europe (0.74; 0.53-1.00); Southern Europe (0.86; 0.77-0.97); former USSR and Baltic States (1.26; 0.73-2.02)	Northeast Asia (0.56; 0.41-0.74); Southeast Asia (0.87; 0.74-1.02); Southern Asia (0.75; 0.59-0.94)	Middle East: (1.10; 0.87-1.39)	South and Central America (0.86; 0.54-1.30)	Africa (0.80; 0.60-1.03)
Canada	Western countries (0.67; 0.65-0.69)		East Asian (0.61; 0.59–0.63); South Asian (0.69; 0.66–0.7)	Middle East (0.63; 0.60-0.67)	Caribbean (0.95; 0.91-1.00) Latin American (0.86; 0.82-0.91)	African (0.80; 0.74-0.85)
Sweden	Germany (1.00; 0.80–1.2); Denmark (0.91; 0.76–1.1) Poland (0.96; 0.78–1.2); Finland (1.07; 0.81–1.4) Norway (0.87; 0.56–1.3); Romania (0.13; 0.03–0.52)	Former Yugoslavia (1.31; 1.10–1.6); former Soviet Union (1.41; 0.92–2.1) Czechoslovakia (0.95; 0.58–1.5) Hungary (1.33; 1.02–1.7)	China/Vietnam (1.50; 0.94–2.4)		Chile (0.79; 0.38–1.7)	

**Table 3:** Summary of results from studies that compared mortality of stroke among immigrants with that of the host population according to country of origin.

Host country	Western Europe, Australia, and North America	Eastern and Middle Europe	East and Southeast Asia	Western Asia/Arab countries	Latin America	Africa
Denmark	Western incl. EU 0.95 (0.35-2.54)	Former Yugoslavia (1.00; 0.73-1.36)	Thailand: NA	Afghanistan (0.46; 0.12-1.87); Iraq (0.88; 0.44–1.76); Turkey (1.60; 0.51–5.03)		Somalia (1.46; 0.47–4.56)
Sweden	Finland (≤10 years) (1.61; 1.37–1.90); Finland (≥11 years) (1.18; 1.02–1.36)					
Northern Ireland	England (1.17; 0.93–1.48); Scotland (0.74; 0.46–1.17); Wales (2.71; 1.41–5.21); Republic of Ireland (0.79; 0.62–1.01)					
The Netherlands	Western (1.09; 1.03 -1.17)		Other non-Western (1.50; 1.11-2.01)	Turkish (1.22; 0.85-1.76)	Surinamese (1.29; 1.05-1.57); Antillean/Aruba (1.17; 0.71-1.94)	
Portugal						All Africans (1.79; 1.54–2.08); Cape Verde (2.65; 2.06–3.40); Angola (1.41; 1.10–1.81)
Canada		Caucasian ethnicity (0.89; 0.83–0.95)	Chinese (0.96; 0.79–1.15); South Asian (1.30; 1.05–1.61)			

**Table 4:** Stratified analyses of the pooled HRs according to country/region of origin.

		Random-effects model		Fixed-effects model		Heterogeneity	
Immigrant subgroup	Number of studies	HR (95% CI)	*P*	HR (95% CI)	*P*	*I* ^2^	*P*
Western Europe, Australia, and North America	6	0.83 (0.74–0.94)	0.003	0.70 (0.68–0.72)	<0.001	84.10%	<0.001
Eastern and Middle Europe	4	1.02 (0.86–1.20)	0.831	0.91 (0.86–0.96)	<0.001	87.20%	<0.001
East and Southeast Asia	5	0.85 (0.73–1.00)	0.044	0.72 (0.71–0.74)	<0.001	97.50%	<0.001
Western Asia/Arab countries	5	0.75 (0.64–0.86)	<0.001	0.69 (0.66–0.72)	<0.001	85.70%	<0.001
Latin America	5	1.08 (0.95–1.23)	0.257	0.95 (0.92–0.98)	0.004	89.20%	<0.001
Africa	4	0.89 (0.66–1.19)	0.430	0.89 (0.84–0.94)	<0.001	95.00%	<0.001

**Table 5:** Relative incidence rate of stroke according to participant characteristics at study entry, comparing immigrants vs. the host population (meanwhile, category variables were defined as gender (the ratio of male immigrates vs. male host with female immigrates vs. female host population), age (the ratio of ≤45 y immigrates vs. ≤45 y host with >45 y immigrates vs. >45 y host population), follow-up duration (the ratio of ≤5 y immigrates vs. ≤5 y host with >5 y immigrates vs. >5 y host population), marital status (the ratio of married immigrates vs. married host with unmarried immigrates vs. unmarried host population), income (the ratio of lower income immigrates vs. lower income host with higher income immigrates vs. higher income host population), residence (the ratio of urban immigrates vs. urban host with rural immigrates vs. rural host population), hypertension (the ratio of not suffered immigrates vs. not suffered host with suffered immigrates vs. suffered host population), diabetes (the ratio of not suffered immigrates vs. not suffered host with suffered immigrates vs. suffered host population), and dyslipidemia (the ratio of not suffered immigrates vs. not suffered host with suffered immigrates vs. suffered host population)).

					Heterogeneity	
Covariate parameters	No. of studies	Pooled OR (95% CI)	*P*	Model	*P* value	*I* ^2^
Gender	8	0.98 (0.94–1.02)	0.293	Random	<0.001	99.50%
Age	2	0.40 (0.03–4.97)	0.475	Random	<0.001	100.00%
Follow-up duration	2	0.68 (0.67–0.69)	<0.001	Fixed	0.399	0.00%
Marital status	2	0.85 (0.53–1.39)	0.525	Random	<0.001	99.90%
Income	5	2.13 (1.65–2.76)	<0.001	Random	<0.001	100.00%
Residence	2	4.59 (3.54–5.95)	<0.001	Random	<0.001	99.80%
Current smoking	2	1.69 (0.92–3.09)	0.090	Random	<0.001	99.70%
*Comorbid conditions*						
Hypertension	4	1.30 (1.08–1.57)	0.006	Random	<0.001	100.00%
Diabetes	4	0.85 (0.72–1.01)	0.059	Random	<0.001	99.90%
Dyslipidemia	3	1.41 (0.93–2.15)	0.109	Random	<0.001	100.00%

## Abbreviations

CI: Confidence interval
RR: Relative risk
HR: Hazard ratios
OR: Odds ratios
NA: Not available.
